The article "Tanshinone IIA alleviates cardiac hypertrophy through m6A modification of galectin-3" was published in 2022. Journal: Bioengineered.

# Tanshinone IIA alleviates cardiac hypertrophy through m6A modification of galectin-3

**DOI:** 10.1080/21655979.2022.2031388

**Published:** 2022-02-22

**Authors:** Meiqi Zhang, Yun Chen, Huan Chen, Ye Shen, Lingxiao Pang, Weihua Wu, Zhenfei Yu

**Affiliations:** a Department of Intensive Care Unit, Hangzhou Hospital of Traditional Chinese Medicine (Dingqiao District), Guangxing Affiliated Hospital of Zhejiang Chinese Medical University, Hangzhou, Zhejiang, China; b Department of Emergency Medicine, Zhejiang Provincial People’ s Hospital (People’s Hospital of Hangzhou Medical College), Hangzhou, Zhejiang, China

**Keywords:** Tanshinone IIA, galectin-3, cardiac hypertrophy, N6-methyladenosine, alkB homolog 5, RNA demethylase

## Abstract

Cardiac hypertrophy results from the adaptive response of the myocardium to pressure overload on the heart. Tanshinone IIA (Tan IIA) is the major active compound extracted from *Salvia miltiorrhiza* Bunge, which possesses various pharmacological benefits. In the present study, the effect and mechanism of action of Tan IIA on cardiac hypertrophy were studied. Ang II–induced and transverse aortic constriction (TAC)-induced cardiomyocyte hypertrophy models were used to evaluate the effect of Tan IIA. An adenoviral vector system was utilized to overexpress galectin-3. The results revealed that Tan IIA significantly inhibited Ang II–induced hypertrophy *in vitro* and TAC-induced cardiac hypertrophy *in vivo*. Furthermore, Tan IIA notably inhibited the expression of galectin-3. Rescue experiments indicated that galectin-3 overexpression reversed the effects of Tan IIA, which further validated the interaction between Tan IIA and galectin-3. Additionally, Tan IIA suppressed alkB homolog 5, RNA demethylase (ALKBH5)-mediated N6-methyladenosine (m6A) modification of galectin-3. In summary, the results of the present study indicated that Tan IIA attenuates cardiac hypertrophy by targeting galectin-3, suggesting that galectin-3 plays a critical role in cardiac hypertrophy and represents a new therapeutic target.

## Introduction

Cardiac hypertrophy is a slow and effective compensatory function of the heart to manage abnormal pressure load [1–3]. This compensatory function leads to an increase in cardiomyocyte volume and protein synthesis, proliferation of myocardial stromal cells, and remodeling of the extracellular matrix, which together cause blood deficiency and hypoxia of the myocardial tissue, weakened myocardial contractility, reduced ventricular compliance, and finally, cardiac enlargement and heart failure [4–7]. However, the mechanism underlying myocardial hypertrophy is not clear. Recently, with the development of molecular biology, it has been found that cellular signal transduction plays an important role in the occurrence and development of myocardial hypertrophy [8]. Thus, it is critical to deeply understand the signal transduction occurring in cardiac hypertrophic cells.

The article "Tanshinone IIA alleviates cardiac hypertrophy through m6A modification of galectin-3" was published in 2022. Journal: Bioengineered.

Tanshinone IIA (Tan IIA) is an active component extracted from *Salvia miltiorrhiza*, a traditional Chinese medicine used in labiatrics. It is a diterpenoid quinone compound and constituent of various plant biochemical reactions and biological activities [9–12]. Previous studies have indicated that Tan IIA plays a critical role in preventing platelet aggregation, free radical damage, and arrhythmia as well as reducing the blood viscosity and improving microcirculation [13–16]. Previous studies have also demonstrated the role of Tan IIA in the prevention of cardiac hypertrophy [17]. However, the mechanism underlying this effect of Tan IIA remains to be elucidated.

In the present study, we confirmed the effect of Tan IIA on cardiac hypertrophy and explored its molecular mechanism of action. Results revealed that Tan IIA alleviated hypertrophy *in vitro* and *in vivo*. It was found that Tan IIA mechanistically participated in m6A modification and regulation of galectin-3 expression. These findings revealed new mechanisms involved in the function of Tan IIA and provided novel potential targets for cardiac hypertrophy therapeutics.

## Materials and methods

### Animals and experimental procedures

The experimental protocol was approved by the Ethics Committee of Hangzhou Hospital of Traditional Chinese Medicine. 6–8-week-old male C57BL/6 mice (20–22 g) were divided into five groups: control, transverse aortic constriction (TAC) (n = 6), TAC + Tan IIA 2 mg/kg (n = 6), TAC + Tan IIA 5 mg/kg (n = 6), and TAC + Tan IIA 10 mg/kg (n = 6). The mice were anesthetized with 2% isoflurane and subjected to TAC surgery. With the 26 G blunt needle, a silk suture (6.0) was placed across the aorta to yield an aorta constriction with a diameter of 0.46 mm. All mice were sacrificed with an intraperitoneal injection of pentobarbital (160 mg/kg). The hearts were weighed after washing with phosphate-buffered saline (PBS).

### Echocardiography for mice

Echocardiography of the left ventricles of mice was performed 4 weeks post-TAC using the Vevo 2100 Imaging System (FUJIFILM, VisualSonics Inc.), as previously reported [18].

### Cell culture and Ang II treatment

Rat heart-derived cells (H9c2), obtained from ATCC (Manassas, VA, USA), were incubated in Dulbecco’s Modified Eagle Medium (DMEM)-high glucose supplemented with 10% FBS, 1% penicillin/streptomycin at 37°C with 5% CO_2_. Myocardial cells were incubated with 10^−5^ mol/l of Ang II 37°C for 48 h.

The article "Tanshinone IIA alleviates cardiac hypertrophy through m6A modification of galectin-3" was published in 2022. Journal: Bioengineered.

### Cell transfection

RNA demethylase (ALKBH5) overexpression plasmids, galectin-3 overexpression plasmids, and the negative control were purchased from GenePharm, Shanghai. Cells were transfected using Lipofectamine 2000 (Invitrogen, Carlsbad, CA, USA). 48 h post-transfection, the cell transfection efficiency was measured by quantitative reverse transcription PCR (RT-qPCR).

### Quantitative reverse transcription PCR

mRNA expression was determined as previously described [7]. TRIzol® reagent (Invitrogen) was used for the isolation of total RNA. Reverse transcription of miRNA was conducted using All-in-One^TM^ miRNA First-Strand cDNA Synthesis Kit, and reverse transcription of Mhrt mRNA was conducted using SureScript™ First-Strand cDNA Synthesis Kit. Subsequently, qPCR was performed using All-in-One™ miRNA qRT-PCR Detection Kit. All the kits used for the experiment were purchased from GeneCopoeia (Guangzhou, China). The relative expression was calculated using the 2^−∆∆CT^ method. U6 was the internal control for miR-765, while GAPDH was the housekeeping gene for Mhrt and other mRNAs.

### Western blot

Protein expression was detected as previously described [19]. All kits or reagents for Western blot were obtained from Elabscience (Wuhan, China). The cells were lysed using RIPA lysis, and protein concentration was tested using the BCA Protein Concentration Detection Kit. 10% SDS-PAGE was performed to separate the proteins and then transferred to PVDF membranes by Western blotting. The membranes were blocked for 1.5 h in 5% skim milk. Next, the membranes were incubated with primary antibodies, such as anti-ANP (ab225844, 1: 1000, Abcam, USA), anti-BNP (ab92500, 1: 5000, Abcam, USA), anti-β-MHC (ab170867, 1: 5000, Abcam, USA), anti-galectin-3 (ab209344, 1: 1000, Abcam, USA), and anti-GAPDH (ab9485, 1: 2500, Abcam, USA) overnight at 4°C and then incubated with a secondary antibody (ab6721, 1: 5000, Abcam, USA) for 1 h at room temperature. The protein bands were visualized using an ECL luminous detection solution, and genes were analyzed and normalized to GAPDH.

### Immunofluorescence (IF) staining

After the cells were treated with Ang II and transfected, they were fixed with 4% formaldehyde and permeabilized in 0.5% Triton X-100 for 20 min at room temperature. After washing with PBS, normal goat serum was added into cells for blocking for 30 min. A primary antibody (α-actinin; Abcam) was added to the cells, followed by incubation overnight at 4°C. On the next day, a secondary antibody (Goat Anti-Mouse IgG H&L (Alexa Fluor® 594; Abcam) was added to the cells, followed by incubation for 1 h. Immunofluorescence was detected using a fluorescence microscope (Olympus, Tokyo, Japan) after the cells were cultured with DAPI for 10 min. In total, 100 cells in 3 wells were randomly selected to quantify the surface area using Image-Pro Plus 6.0.

The article "Tanshinone IIA alleviates cardiac hypertrophy through m6A modification of galectin-3" was published in 2022. Journal: Bioengineered.

### RNA total m6A quantification

Total RNA was extracted from THP-1 and U937 macrophages, followed by mRNA purification. An m6A RNA Methylation Quantification Kit (Colorimetric) (ab185912, Abcam, USA) was used to determine the total level of m6A in treated cells. Subsequently, the m6A content was quantified at a wavelength of 450 nm.

### Methylated RNA immunoprecipitation (MeRIP) assay

The purified mRNA fragments were incubated with the m6A antibody for immunoprecipitation using the Magna MeRIP™ m6A kit (#17–10,499, Merck Millipore, Germany). Briefly, 30 μg of the total RNA was collected and mixed with the MeRIP reagent. The previously resuspended Magna ChIP protein A/G Magnetic Beads were conjugated with anti-m6A (MABE1006, Merck Millipore, Germany) or normal mouse anti-IgG antibodies (CS200621, A&D Technology, Japan) overnight at 4°C. Finally, the magnetic beads were eluted from the complex, and the RNA level was quantified using RT-qPCR.

### Statistical analysis

All experiments were repeated at least three times, and the data was represented as mean ± standard deviation (SD). GraphPad Prism 6.0 software (GraphPad, CA, USA) was used for the analysis. Significant differences were analyzed according to Student’s t-test (between two groups) and one-way ANOVA (in multiple groups). *P* < 0.05 was considered statistically significant.

## Results

In this study, Tan IIA played a beneficial role in the development of cardiac hypertrophy. Tan IIA suppressed m6A modification of galectin-3 via downregulating ALKBH5, which suppressed the development of cardiac hypertrophy.

### Tan IIA attenuated cardiac hypertrophy *in vitro*

The structure of Tan IIA is shown in Figure 1(a). First, Ang II was used to induce an *in vitro* cardiac hypertrophy model. Different concentrations of Tan IIA were administered to H9c2 cells. It was observed that 200 and 400 μM of Tan IIA inhibited the viability of H9c2 cells (Figure 1(b)). Thus, we chose 25, 50, and 100 μM of Tan IIA for further studies. IF staining of α-actin was performed to calculate the surface area of H9c2 cells. Furthermore, Ang II administration notably increased the size of H9c2 cells, while 25, 50, and 100 μM of Tan IIA reduced it (Figure 1(c)). In addition, qPCR and Western blot results indicated that Ang II treatment significantly increased the mRNA and protein expression level of ANP, BNP, and β-MHC. Tan IIA (25, 50, and 100 μM) notably inhibited this elevation in a dose-dependent manner (Figure 1(d,e)). These results indicate that Tan IIA can alleviate Ang II–induced cardiac hypertrophy.

The article "Tanshinone IIA alleviates cardiac hypertrophy through m6A modification of galectin-3" was published in 2022. Journal: Bioengineered.

**Figure 1.** Effects of Tan IIA on Ang II–induced hypertrophy of H9c2 cells. (a) Molecular structure of Tan IIA. (b) MTT assay was performed to measure the inhibition rate of Tan IIA on the H9c2 cells. (c) Immunofluorescence staining of α-actin was performed to evaluate the surface area of H9c2 cells. (d, e) qPCR and Western blot were used to detect the expression of ANP, BNP, and β-MHC. ***P < 0.001 vs. control group, ^#^*P* < 0.05 vs. Ang II group, ^##^*P* < 0.01 vs. Ang II group, ^###^*P* < 0.001 vs. Ang II group.

### Tan IIA attenuated cardiac hypertrophy in vivo

TAC was used to establish an *in vivo* cardiac hypertrophic model. The results of HE staining indicated that TAC treatment significantly increased the size of the cardiomyocytes while Tan IIA administration reduced it (Figure 2(a)). In addition, we evaluated the cardiac function using echocardiography. It was shown that TAC increased the left ventricular end-diastolic and end-systolic diameters (LVEDd and LVESd, respectively) and decreased the LV fractional shortening and LV ejection fraction (LVFS and LVEF, respectively). In contrast, 25, 50, and 100 μM of Tan IIA significantly reduced LVEDd and LVESd, while increasing the LVFS and LVEF (Figure 2(b–e)). In addition, heart weight/tibia length (HW/TL) was calculated. TAC increased the HW/TL of mice, while 50 and 100 μM of Tan IIA significantly reduced it (Figure 2(f)).

**Figure 2.** Effects of Tan IIA on cardiac hypertrophy *in vivo*. (a) HE staining was performed to evaluate the pathological changes of myocardial structure. (b–e) Echocardiography was used to evaluate the cardiac function. (f) HW/TL was calculated in each group. **P < 0.05 vs. control group, ***P < 0.001 vs. control group, ^#^P < 0.05 vs. Ang II group, ^##^*P* < 0.01 vs. Ang II group, ^###^*P* < 0.001 vs. Ang II group.

### Tan IIA inhibited the expression of galectin-3

Increasing studies have reported that galectin-3 is involved in the progression of cardiac hypertrophy. Therefore, we evaluated the expression of galectin-3 in the mechanism of Tan IIA action. The qPCR and Western blot results indicated that the expression of galectin-3 was significantly downregulated in H9c2 cells treated with Tan IIA and in the myocardium of TAC mice (Figure 3(a–d)).

**Figure 3.** Effects of Tan IIA on the mRNA and protein expression of galectin-3 in H9c2 cells. qRT-PCR (a) and Western blot analysis (b) were performed to examine the expressions of galectin-3 in each group. ***P < 0.001 vs. control group, ^#^P < 0.05 vs. Ang II group, ^##^*P* < 0.01 vs. Ang II group, ^###^*P* < 0.001 vs. Ang II group, ^&&^*P* < 0.01 vs. Tan IIA group, ^&&&^*P* < 0.001 vs. Tan IIA group.

The article "Tanshinone IIA alleviates cardiac hypertrophy through m6A modification of galectin-3" was published in 2022. Journal: Bioengineered.

### Galectin-3 reversed the effect of Tan IIA on cardiac hypertrophy

Rescue experiments were performed to elucidate the role of galectin-3 in cardiac hypertrophy. Results indicated that the transfection of pc-DNA3.1/galectin-3 significantly promoted the expression level of galectin-3 (Figure 4(a)). Evaluation of cardiomyocyte size and expression of hypertrophic genes demonstrated that galectin-3 overexpression reversed the protective effect of Tan IIA on cardiac hypertrophy *in vitro* (Figure 4(b–d)).

**Figure 4.** Galectin-3 overexpression reverses the effect of Tan IIA on cardiac hypertrophy. qPCR was used to detect the expression of galectin-3 in H9c2 cells. (b) Immunofluorescence staining of α-actin was performed to evaluate the surface area of H9c2 cells. (c, d) qPCR and Western blot were used to detect the expression of ANP, BNP, and β-MHC. **P < 0.01 vs. control group, ***P < 0.001 vs. control group, ^##^P < 0.01 vs. Ang II group, ^###^*P* < 0.001 vs. Ang II group, ^&&^*P* < 0.01 vs. Ang II group, ^&&&^*P* < 0.001 vs. Ang II group.

### Tan IIA inhibited m6A modification and expression of galectin-3

The above mentioned findings revealed that Tan IIA could attenuate cardiac hypertrophy by inhibiting galectin-3 expression. However, the regulation mechanism of galectin-3 expression by Tan IIA remains unclear. We found that Ang II treatment inhibited the total m6A modification of H9c2 cells while Tan IIA treatment promoted it (Figure 5(a)). Moreover, the MeRIP assay indicated that the m6A modification of galectin-3 was also promoted by Ang II treatment, while the same was inhibited by Tan IIA (Figure 5(b)). Subsequently, the expression levels of RNA methylase (METTL3, METTL14, and WTAP) and demethylase (FTO, AlkB homolog H5 [ALKBH5]) were evaluated. It was found that Tan IIA significantly suppressed the expression of ALKBH5 (Figure 5(c)). To confirm the participation of ALKBH5 in the m6A modification of galectin-3, ALKBH5 silencing was carried out. ALKBH5 knockdown reversed the inhibitory effect of Ang II on m6A modification, while ALKBH5 overexpression inhibited m6A modification of galectin-3 (Figure 5(d)). ALKBH5 could also reverse the inhibitory effect of Tan IIA on m6A modification of galectin-3 (Figure 5(e)). The qPCR and Western blot results indicated that ALKBH5 reversed the inhibitory effect of Tan IIA on the expression of galectin-3 (Figure 5(f–h)). Furthermore, we evaluated the stability of galectin-3 mRNA. Notably, Ang II promoted the stability of galectin-3 mRNA, which could be reversed by Tan IIA. ALKBH5 overexpression reversed this effect of Tan IIA (Figure 5(i)).

The article "Tanshinone IIA alleviates cardiac hypertrophy through m6A modification of galectin-3" was published in 2022. Journal: Bioengineered.

**Figure 5.** Tan IIA regulates ALKBH5-mediated m6A modification of galectin-3. The total m6A content of H9c2 cells was detected. (b) MeRIP assay was performed to detect the m6A modification of galectin-3. (c) qPCR was used to detect the expression of methylases and demethylases. (d, e) MeRIP assay was performed to detect the m6A modification of galectin-3. (e–h) qPCR and Western blot were used to the expression of galectin-3. (f) qPCR was performed to detect the stability of galectin-3 mRNA. ***P < 0.001 vs. control group, ^##^*P* < 0.01 vs. Ang II group, ^&^*P* < 0.05 vs. Ang II group, ^&&^*P* < 0.01 vs. Ang II group.

### ALKBH5 reversed the effect of Tan IIA on cardiac hypertrophy

Rescue experiments were performed to elucidate the role of ALKBH5 in cardiac hypertrophy. Quantification of cardiomyocyte size and the expression of hypertrophic genes demonstrated that ALKBH5 overexpression reversed the protective effect of Tan IIA on cardiac hypertrophy *in vitro* (Figure 6(a–e)).

**Figure 6.** ALKBH5 reverses the effect of Tan IIA on cardiac hypertrophy. (a) Immunofluorescence staining of α-actin was performed to evaluate the surface area of H9c2 cells. (b–e) qPCR and Western blot were used to detect the expression of ANP, BNP, and β-MHC. ***P < 0.001 vs. control group, ^##^*P* < 0.01 vs. Ang II group, ^###^*P* < 0.001 vs. Ang II group, ^&&^*P* < 0.01 vs. Ang II group.

## Discussion

Previous studies have confirmed the role of Tan IIA in the inhibition of cardiac hypertrophy. The mechanism underlying this effect of Tan IIA is complicated. For instance, Tan IIA alleviates cardiac hypertrophy via inhibiting calcineurin/NFATc3 or Cys-c/Wnt signaling [20,21]. It also attenuates Leu27IGF-II-induced hypertrophy through estrogen receptor-mediated activation of the AKT pathway [22]. Through the current study, we found that Tan IIA inhibited Ang II–induced cardiomyocyte hypertrophy, which is consistent with the findings of earlier studies [23].

Mechanistically, we demonstrated that Tan IIA could inhibit the expression of galectin-3, which has not been reported to date. In our previous study, we confirmed that galectin-3 mediated the inhibitory effect of miR-27b on cardiac hypertrophy [18]. Galectin-3, which plays a critical role in the progression of various cardiovascular diseases, is unique since it is the only member of the galectin family with an extended N-terminal domain [24]. It promotes lipid metabolism and induces cardiac remodeling *via* suppressing the Akt signal pathway [25]. Galectin-3 is also a potential biomarker to predict arrhythmia risk or antiarrhythmic prophylaxis [26]. Besides, the loss of galectin-3 may delay the hypertrophic response after pressure overload on the heart, confirming the role of galectin-3 in mediating cardiac hypertrophy [27].

The article "Tanshinone IIA alleviates cardiac hypertrophy through m6A modification of galectin-3" was published in 2022. Journal: Bioengineered.

In the present study, we reported that Tan IIA inhibited the mRNA and protein expression of galectin-3 to exert its effect on cardiac hypertrophy. Furthermore, we speculated how Tan IIA inhibited the expression of galectin-3.

Several recent studies confirmed that m6A methylation was closely related to the progression of cardiac hypertrophy [28]. Methylase METTL3 participates in regulating cardiac homeostasis and hypertrophy [29]. PiRNA CHAPIR promotes cardiac hypertrophy through METTL3-mediated m6A modification of Parp10 mRNA [30]. As the most common regulation of RNA methylation, m6A is co-regulated by methyltransferase complexes (METTL3, METTL14, and WTAP), demethylase (FTO and ALKBH5), and their corresponding readers (YTHDF1/2/3, YTHDC1) [31–33]. In the present study, we confirmed that Tan IIA treatment could reverse the effect of Ang II on the reduction of m6A content in H9c2 cells. In addition, Tan IIA promoted the m6A modification of galectin-3. Subsequently, we investigated which methylase or demethylase may be involved in this effect of Tan IIA. qPCR results indicated that the expression of ALKBH5 was significantly downregulated after Tan IIA treatment in H9c2 cells. We performed a rescue experiment to confirm whether Tan IIA exerts its effect *via* regulating ALKBH5 expression. The results indicated that Tan IIA promotes the m6A modification of galectin-3 *via* inhibiting ALKBH5 expression. The m6A modification inhibits the stability of galectin-3 mRNA. Thus, Tan IIA inhibits the expression of galectin-3. We revealed the role of Tan IIA in galectin-3 and m6A modification as well as the role of ALKBH5 in cardiac hypertrophy. However, the precise mechanisms involving Tan IIA and m6A modification need further elucidation. For instance, the m6A reader that recognizes the modification and influences the stability of galectin-3 mRNA will be studied in our future work.

## Conclusion

In conclusion, this study investigated the therapeutic effects of Tan IIA on myocardial hypertrophy. We revealed, for the first time, that Tan IIA could prevent cardiac hypertrophy, mediated by m6A modification and the regulation of galectin-3 expression. These findings provide a foundation for the potential development of Tan IIA as a therapeutic drug for cardiac hypertrophy.

## Highlights

1. Tanshinone IIA suppressed cardiomyocyte hypertrophy *in vitro*.
2. Tanshinone IIA suppressed the protein expression of galectin-3.
3. Tanshinone IIA inhibited the mRNA expression of galectin-3 via suppressing ALKBH5 mediated m6A modification of galectin-3.
4. Tanshinone IIA suppressed cardiomyocyte hypertrophy *in vivo*.
